The article "miR-4780 Derived from N2-Like Neutrophil Exosome Aggravates Epithelial-Mesenchymal Transition and Angiogenesis in Colorectal Cancer" was retracted in 2023. Reasons: signs of a paper mill; suspected computer-generated content; unreliable results or conclusions; lack of ethics approval or compliance.

# miR-4780 Derived from N2-Like Neutrophil Exosome Aggravates Epithelial-Mesenchymal Transition and Angiogenesis in Colorectal Cancer

**DOI:** 10.1155/2023/2759679

**Published:** 2023-08-04

**Authors:** Liang Wang, Yuqiang Shan, Sixin Zheng, Jiangtao Li, Peng Cui

**Affiliations:** ^1^Department of Gastrointestinal and Anal Surgery, Affiliated Hangzhou First People's Hospital, Zhejiang University School of Medicine, Hangzhou, China; ^2^Department of Gastrointestinal Surgery, Changzhi People's Hospital, Affiliated Hospital of Changzhi Medical College, Changzhi, China

## Abstract

Despite significant advances in diagnostic methods and treatment strategies, the prognosis for patients with advanced colon cancer remains poor, and mortality rates are often high due to metastasis. Increasing evidence showed that it is of significant importance to investigate how the tumor microenvironment participates in the development of colorectal cancer (CRC). In this manuscript, neutrophils were sequentially stimulated with all-trans retinoic acid and transforming growth factor-*β* in turn to induce the neutrophil polarization. Differentially expressed miRNA in neutrophil exosomes have been sequenced by microarray profile, and the effect of N2-like neutrophil-derived exosomal miR-4780 on epithelial-mesenchymal transition (EMT) and angiogenesis was investigated. In our results, we found that neutrophils were enriched in CRC tumor tissue and that CD11b expression correlated with tumor site and serous membrane invasion. At the same time, we demonstrated that internalization of N2 exosomes exacerbated the viability, migration, and invasion of CRC cell lines and inhibited apoptosis. To further investigate the molecular mechanism, we analyzed the miRNA expression profile in the N2-like neutrophils, which led to the selection of hsa-miR-4780 for the subsequent experiment. The overexpression of miR-4780 from N2-like neutrophil-derived exosomes exacerbated EMT and angiogenesis. Moreover, miR-4780 can regulate its target gene SOX11 to effect EMT and angiogenesis in CRC cell lines. CRC with liver metastasis model also validated that aberrant expression of miR-4780 in N2-like neutrophil exosomes exacerbated tumor metastasis and development of tumor via EMT and angiogenesis. In conclusion, our current findings reveal an important mechanism by which mR-4780 from N2-like neutrophil exosomes exacerbates tumor metastasis and progression via EMT and angiogenesis.

## 1. Introduction

Colorectal cancer (CRC) is one of the most prevalent tumors worldwide [1]. Although considerable progresses have been made in diagnosing approaches and therapeutic strategies for CRC, the prognosis for patients with advanced stage is still poor due to the metastases, and usually distant metastasis contributes to high mortality [2]. Therefore, it is crucial to investigate the occurrence and development of metastases in CRC. Increasing evidence has revealed that tumor microenvironment (TME) also participates in cancer pathogenesis besides genetic alterations and dysregulation of intracellular pathways [3–5]. TME is associated with tumor generation, development, and metastasis [6, 7]. It mainly contains various immune cells and tumor-related stromal fibroblasts, among which immune cells are one of the main components in the TME [8]. During the carcinogenesis, the change in microenvironment toward an inflammatory milieu and contributes to tissue remodeling and tumor progression; the dynamic tumor interaction with TME is therefore associated with the regulation of neoangiogenesis, the supply of growth factors and cytokines, and remodeling of the extracellular matrix (ECM), as well as immune escape and drug resistance [9–12]. It has become evident that stromal cells also contribute to the polarization and activation of immune cells within TME [13–15].

The article "miR-4780 Derived from N2-Like Neutrophil Exosome Aggravates Epithelial-Mesenchymal Transition and Angiogenesis in Colorectal Cancer" was retracted in 2023. Reasons: signs of a paper mill; suspected computer-generated content; unreliable results or conclusions; lack of ethics approval or compliance.

Neutrophils are regarded as the most abundant circulating leucocytes to participate in the regulation of innate and adaptive immune systems [16]. As a critical role in TME, neutrophils were now found as active participants in the development, growth, and progression of various tumors [17, 18]. Classically, neutrophils induce phagocytosis and release lysozyme and product of reactive oxygen species to protect the body from microbial infection and eliminate pathogens [19–21]. In the context of TEM, neutrophils have been proved can be polarized towards two distinct populations and play a dual role in tumor suppressive factor and tumor promotive factor [22]. In the early stage, neutrophils are recruited to the malignant site and suppress carcinogenesis via cytotoxic and immune response, which is defined as N1-like neutrophils. However, with tumors developed to intermediate and advanced stages, neutrophils are accumulated in the tumor matrix [23]. Attributed to factors encountered in TME, the changes of neutrophils in phenotype and function occur, which are regarded as N2-like neutrophils [24]. Interestingly, the considerable plasticity between tumor-suppressive and-supportive neutrophils is regulated by polarization induced by transforming growth factor (TGF)-*β* and interferon-*β* signaling [25, 26]. Tumor-associated neutrophils (TANs) can secrete multiple factors and assist in the growth, migration, invasion, and angiogenesis in various cancer cells and are proven to be associated with immune escape and drug resistance [27]. Tohme et al. [28] proved that neutrophils secrete HMGB1 during NETosis, thereby promote the adhesion, proliferation, migration, and invasion. Exosomes are referred to as 40–150 nm membrane vesicles with lipid membranes [29]. Exosomes can be derived by numerous types of cells (i.e., dendritic cells, reticulocytes, tumor cells, B cells, T cells, mast cells, epithelial cells, and BMSCs) and released into the extracellular environment [30–32]. However, the function of N2-like neutrophils derived exosome exerts on epithelial-mesenchymal transition (EMT) and angiogenesis in CRC is unrevealed yet.

The article "miR-4780 Derived from N2-Like Neutrophil Exosome Aggravates Epithelial-Mesenchymal Transition and Angiogenesis in Colorectal Cancer" was retracted in 2023. Reasons: signs of a paper mill; suspected computer-generated content; unreliable results or conclusions; lack of ethics approval or compliance.

In this study, differentially expressed miRNA in neutrophils-derived exosomes have been sequenced by microarray profile, and EMT-associated miRNA, miR-4780, was selected, and the effect of N2-like neutrophils-derived exosomal miR-4780 on EMT and angiogenesis was investigated. In conclusion, N2-like neutrophils-derived exosomal miR-4780 aggravates EMT and angiogenesis in CRC.

## 2. Material and Methods

### 2.1. Clinical Data

Primary CRC tissues and their corresponding para-cancerous tissue from 30 patients diagnosed with CRC (16 males and 14 females, mean age at 63.27 ± 9.93) were harvested from the First Affiliated Hospital of Kunming Medical University from 2017 to 2019. Inclusion criteria: (i) patients with the primary CRC; (ii) patients with complete clinical data; (iii) none of the patients had undergone radiotherapy and molecular targeted therapy before surgery; (iv) patients aged 36–82 years. Exclusion criteria included: (i) patients with nonprimary CRC and combined with other primary tumors; (ii) patients with gastrointestinal diseases, acute or chronic infections; (iii) patients with combined serious diseases of liver, cardiovascular, hematological system, and/or kidney; (iv) patients with psychiatric disorders. This study was approved by the ethics review committee of Affiliated Hangzhou First People's Hospital, Zhejiang University School of Medicine (No. 2022-59-01). All corresponding participants were fully informed the usage and data retrieval and provided their written informed consent to participate before the acquisition of specimens. The study does not contain information or images that could lead to the identification of any involved patient or that could violate any personal rights. The clinicopathologic parameters are shown in *Supplementary 1*.

### 2.2. Immunohistochemistry Staining

Immunohistochemistry staining (IHC) was performed as previously described [33]. In brief, the paraffin sections were deparaffinized and rehydrated. The slides were incubated with the preimmune serum to eliminate nonspecific staining, then immersed into methanol containing 0.3% to inactivate endogenous peroxidase at room temperature for 30 min. The sections were stained with primary antibody to CD66b (1 : 500, ab197678, Abcam, UK), CD11b (1 : 700, ab197678, Abcam, UK) overnight at 4°C. Then slides were exposed to appropriate secondary antibody at 37°C for 30 min using EnVisionTM + Dual Link System-HRP (Dako North America, Inc. Carpinteria, CA 93013, USA). DAB (3,3-diaminobenzidine) and chromogen solution were used for color reaction enhancement. Hematoxylin was used to counterstain the slides. Images were acquired by laser scanning confocal microscopy (LSM710, Carl Zeiss, Germany) and analyzed using Image-Pro Plus 6.0.

The article "miR-4780 Derived from N2-Like Neutrophil Exosome Aggravates Epithelial-Mesenchymal Transition and Angiogenesis in Colorectal Cancer" was retracted in 2023. Reasons: signs of a paper mill; suspected computer-generated content; unreliable results or conclusions; lack of ethics approval or compliance.

### 2.3. Cell Culture of Colorectal Cancer Cell Lines

Human CRC cell line SW480 (BNCC100604, BeNa culture collection, China) and COLO205 (ml039630, mlBio, China) were used from further investigations. All the cells were cultured in RPMI 1640 (Hyclone, USA) containing 10% fetal bovine serum (FBS) (Hangzhou Sijiqing Biotech, Co. Ltd. China) and 1% Penicillin/Streptomycin in a humidified 5% CO_2_ at 37°C. SOX11 expression vector pcDNA3.1 and pcDNA-SOX11 were purchased from the Genepharma, China. The pcDNA3.1 and pcDNA-SOX11 were transfected to SW480 and COLO205 via Lipofectamine 2000 agent (Invitrogen, Carlsbad, CA, USA) in accordance with the manufacturer's protocol. About 48 hr after transfection, fresh RPMI 1640 medium with 10% FBS was added.

### 2.4. Neutrophil Polarization and Verification

Human myeloid leukemia cell line NB-4 cells were purchased from ATCC (Bioleaf, China) and induced neutrophil polarization according to the previous manuscript [34]. In brief, 100 mg all-trans retinoic acid (ATRA, R2625, Sigma, MO, USA) powder was dissolved in 10 mL dimethyl sulfoxide under aseptic conditions to prepare a storage solution at a concentration of 33.2 mM/L. NB-4 cell line was cultured in RPMI-1640 culture medium containing 10% FBS in the presence of 5% CO_2_ at 37°C. About 1 *μ*mol/L ATRA was utilized to differentiate NB-4 to neutrophil-like cells for 4 or 5 days. The morphology of differentiated neutrophil-like NB-4 cells was observed under an optical microscope and verified by Wright's stain. The differentiated neutrophil-like NB-4 cells were separated into two groups, N0-like neutrophil (differentiated neutrophil-like NB-4 cells were left untreated) and N2-like neutrophil. In N2-like neutrophil group, neutrophil-like NB-4 cells were induced to N2-like polarization by TGF-*β* under selected concentration for 24 hr according to different polarity disposal conditions of neutrophils [25]. miR-4780 inhibitor and its corresponding nonspecific vector were synthesized (Ribo Bio, China) and transfected into neutrophils, according to the manuscript.

The article "miR-4780 Derived from N2-Like Neutrophil Exosome Aggravates Epithelial-Mesenchymal Transition and Angiogenesis in Colorectal Cancer" was retracted in 2023. Reasons: signs of a paper mill; suspected computer-generated content; unreliable results or conclusions; lack of ethics approval or compliance.

### 2.5. Detection of Neutrophil Activation

To screen the concentration of TGF-*β* on N2-like polarization, the proportion of CD11b and CD66b was detected by flow cytometer. ATRA-treated neutrophil-like NB-4 cells were collected, and TGF-*β* in different concentrations was applied. The 5 *μ*L antibody to CD11b (ab24874, Abcam, UK) and CD66b (ab275587, Abcam, UK) was added, and cell fluorescence was detected under flow cytometry.

### 2.6. The Extraction and Uptake of Neutrophil-Derived Exosomes

Exosome isolation was performed via Exosome extraction reagent in the ratio of 1 : 4 (Ribo, China). About 300 mL supernatants of neutrophils were centrifuged at 2,000 *g* for 30 min to remove the precipitation. Then the supernatants containing exosomes were first concentrated using a 100 kDa ultrafiltration Vivaflow 200 module to 10–15 mL and to a final volume of between 0.5 and 1 mL by a 100 kDa ultracentrifuge tube (3,000 *g* × 30 min). Next, exosomes were precipitated by adding exosome extraction reagent at the ratio of 1 : 4 and incubated overnight at 4°C. Then the exosome precipitation was obtained by centrifugation at 1,500 *g* for 30 min, resuspended in phosphate-buffered saline (PBS). Exosome protein content was measured using bicinchoninic acid (BCA) protein assay kit (Thermo Fisher Scientific, CN). The isolated exosomes were observed and identified by transmission electron microscopy (TEM) [35].

About 60 *μ*g of isolated exosomes were incubated with 1 mL PKH-67 green fluorescent dye for 5 min (1 × 10-3 mM, Sigma Aldrich, Germany) and washed to remove excess dye using 100 kDa filter. Then, the labeled exosomes were incubated with the recipient, namely, CRC cell lines COLO205 and SW480, respectively, for 48 hr, and then the recipients were stained with DAPI and photographed using a laser-scanning confocal microscope.

### 2.7. Cell Proliferation and Apoptosis

The viability of CRC cell lines was evaluated using Cell Counting Kit-8 (CCK-8, Dongren Chemical Technology Co., Ltd., Shanghai, China), according to the manufacturer's instructions. Cells were incubated with CCK-8 reagent for 1 hr, and absorbance at 450 nm was measured with a microplate reader (Tecan, Männedorf, Switzerland).

For flow cytometry, cell was fixed with precooled 70% alcohol for 24 hr, washed with PBS, and then incubated with propidium iodide (PI) (Dongren Chemical Technology Co., Ltd, Shanghai, China) under dark conditions at 4°C. Cell cycle stages were detected by a flow cytometer (Partec GmbH, CyFlow Space). Cell apoptosis was detected using the Annexin V-FITC/PI staining. 100 *μ*L of 1 × 10^6^ cells/mL cell suspension was added into 5 mL of Annexin V-FITC (Partec GmbH, CyFlow Space) and 10 *μ*L of PI, and the culture was incubated at room temperature for 15 min and washed twice with PBS. Cell apoptosis was analyzed using a flow cytometer at an excitation wavelength of 488 nm.

The article "miR-4780 Derived from N2-Like Neutrophil Exosome Aggravates Epithelial-Mesenchymal Transition and Angiogenesis in Colorectal Cancer" was retracted in 2023. Reasons: signs of a paper mill; suspected computer-generated content; unreliable results or conclusions; lack of ethics approval or compliance.

### 2.8. Migration and Invasion Assay

Cell wound healing assay was used to detect the ability of cell migration. When cells were 80%–90% confluent, the cell monolayer was scraped with a sterile 200 *μ*L pipette tip. After being incubated for 24 hr, the cells were fixed, and images were taken. The migration distance and mobility were calculated using ImageJ (version 1.80, National Institutes of Health, Bethesda, MD, USA).

For cell invasion assay, cell suspension (1 × 10^4^ cells) in FBS-free medium was plated in the upper chamber coated with Matrigel (Corning, Costar, Corning, NY, USA) and incubated for 24 hr. After incubation, cells that had invaded the lower chamber were fixed with 4% paraformaldehyde and stained with crystal violet solution (Beyotime Biotechnology, China). The number of cell invasion in five random fields were counted using ImageJ.

### 2.9. Tube Formation

Human umbilical vein endothelial cells (HUVECs, ATCC, VA, USA, cat. No. PCS-100-010) were cultured with CRC cell lines in a ratio of 3 : 1 [36]. Matrigel was diluted to 5 mg/mL with serum-free Dulbecco's Modified Eagle Medium and plated at 37°C for 30 min to harden the Matrigel. Then, 1.5 × 10^4^ cells were inoculated in 96-well plates on the pre-coated Matrigel for 6 hr at 37°C. Four random fields were taken at capillary-like structures were counted with ImageJ.

### 2.10. Quantitative Polymerase Chain Reaction (qPCR)

TRIzol reagent (Invitrogen, USA) was used to extract the total RNA from exosomes or CRC cell lines COLO205 and SW480. Nanodrop ND-1000 (Nanodrop, DE, USA) was employed to verify the quality and quantity of extracted RNA. The integrity of RNA was assessed by standard denaturing agarose gel electrophoresis. PCR was performed using cDNA and SYBR Green Real-Time PCR Master Mixes (Thermo Fisher Scientific, USA) with initial denaturation at 95°C for 1 min, 35 cycles of denaturation at 95°C for 1 min, annealing at 60°C for 2 min, and extension for 30 s, at 72°C. Primers were designed and validated by Ribo Co. Ltd. Results of the log-linear phase of the growth curve were analyzed, and relative quantification was performed using the 2^−*ΔΔ*Ct^ method with *β*-actin and GAPDH as a housekeeping gene. Each experiment was repeated independently three times.

### 2.11. Western Blot

Cells and liver tissues from liver metastasis model were collected and lysed in radio immunoprecipitation assay lysis buffer (containing 0.01% phenylmethanesulfonyl fluoride, 150 nmol/L Tris (pH = 8), 0.1% SDS, 0.2% ethylenediaminetetraacetic acid, 1% Triton X-100, 1% sodium deoxycholate). BCA protein assay kit (KeyGen Biotech, China) was used to detect the protein concentration. The total protein samples were separated by sodium dodecyl sulfate-polyacrylamide gel electrophoresis and transferred to polyvinylidene fluoride membranes. The membranes were blocked using 5% skimmed milk at room temperature for 2 hr and then were probed with primary antibodies overnight at 4°C. Primary antibodies are listed in Table 1. After washing by TBS-T, membranes were incubated with horseradish peroxidase-conjugated secondary antibodies for 2 hr at room temperature. Enhanced chemiluminescence assay was used and captured through Imager. The optical density of the bands was analyzed using NIH ImageJ software.

The article "miR-4780 Derived from N2-Like Neutrophil Exosome Aggravates Epithelial-Mesenchymal Transition and Angiogenesis in Colorectal Cancer" was retracted in 2023. Reasons: signs of a paper mill; suspected computer-generated content; unreliable results or conclusions; lack of ethics approval or compliance.

### 2.12. Enzyme-Linked Immunosorbent Assay (ELISA)

The concentrations of CXCL10, IL-12, IL-10, and CCL2 were measured via ELISA [36]. According to the instructions of ELISA Kit, the supernatant was collected by centrifugation homogenate (5,000 rpm for 15 min at 4°C). The activities of CXCL10, IL-12, IL-10, and CXCL2 were determined by ELISA Kit. Quantification of ELISA results was performed at 450 nm using an ELISA plate reader (Spectra Max M5, Molecular Devices, USA).

### 2.13. Colorectal Cancer with Liver Metastasis Model

CRC with liver metastasis model was established via splenic injection model (SIM) [37] as described before. In brief, 50 athymic nude mice (BALA/c mice) were sterilized with 83% alcohol after inhalation anesthesia. A left lateral flank incision was made, and peritoneum was opened (at an approximate 8 mm length) to expose the spleen. CRC cells (2 × 10^6^/100 *μ*L) were injected slowly into the splenic parenchyma. After recovering from anesthesia, mice were returned to the cage. Fifteen days after SIM establishment, 200 *μ*L exosomes were intraperitoneally injected. *In vivo* live imaging was conducted twice weekly to monitor metastatic spread. Twenty-eight days after model establishment, mice were euthanized by dislocated cervical vertebrae, and liver tissue samples were collected and further examined by Western blot, IHC, qPCR, and immunofluorescence. All experimental procedures involved animals were conducted in accordance with the guidelines of the Animal Experimental Center of Zhejiang University School of Medicine and approved by the ethics committee of Zhejiang University School of Medicine (No. 22476); animals underwent all procedures under anesthesia, and every effort was made to minimize pain and death.

### 2.14. Immunofluorescence

Sections (5 *μ*m) were stained by Immunofluorescence. Specifically, sections were washed with PBS and fixed with 4% paraformaldehyde for 20 min at room temperature and then blocked in 5% goat serum for 1 hr and labeled with primary antibodies against ZO1 (61-7300, Thermo Fisher, China, 1 : 100) and vimentin (5741 S, CST, China, 1 : 100) overnight at 4°C. After that, sections were incubated in secondary antibodies for 30 min at 37°C. Then, coverslips were sealed using Prolong Gold antifade reagent with DAPI (Invitrogen, Carlsbad, CA). Images were acquired by laser scanning confocal microscopy (LSM710, Carl Zeiss, Germany) and analyzed using Image-Pro Plus 6.0.

The article "miR-4780 Derived from N2-Like Neutrophil Exosome Aggravates Epithelial-Mesenchymal Transition and Angiogenesis in Colorectal Cancer" was retracted in 2023. Reasons: signs of a paper mill; suspected computer-generated content; unreliable results or conclusions; lack of ethics approval or compliance.

### 2.15. Statistics Analysis

Results were performed as mean value ± standard deviation (SD) and analyzed with Graph-Pad Prism (GraphPad Software, ver. 9.0.0, San Diego, CA). Statistical analyses were performed using one-way analysis of variance, followed by Turkey's post-test. Pearson's correlation analysis was performed to assess the relationship between CD66b and CD11b expression and clinicopathological status by SPSS statistical software (version 22.0, IBM, SPSS, USA). All experiments for cell culture were performed independently at least three times and in triplicate each time. Differences with *p* < 0.05 were considered statistically significant.

## 3. Results

### 3.1. Neutrophils Accumulation is Associated with Colorectal Cancer Metastasis

To evaluate the distribution of neutrophils in TME, gene set enrichment analysis was performed via cancer immunome database (TCIA, https://tcia.at/home). The result revealed that neutrophils are relatively enriched in liver hepatocellular carcinoma, stomach adenocarcinoma, bladder cancer, lung adenocarcinoma, and CRC (Figure 1(a)). The fraction of immune cell profile in TME of CRC showed that neutrophils (32%), M1-like macrophage (27%), and M2-like macrophage (11%) are the most infiltrated immune cells in CRC (Figure 1(b)). Also, the results of immunohistochemistry showed the expression of neutrophils markers CD66b and CD11b located in stroma. Consistently, it is observed that the expression of CD66b and CD11b was increased in CRC tissues compared with para-cancerous tissues (Figure 1(c)–1(f)), which indicated that neutrophils were accumulated in CRC tissues. Also, as shown in Table 2, the CD11b expression is correlated with tumor site and the presence of invasion of serosa, while no correlation was found between CD66b and clinicopathologic parameters.

### 3.2. Exosome Derived from Neutrophils Aggravated Aggressive Behavior of CRC

To further investigate the effect of exosome derived from neutrophils on CRC aggressive behavior, we first induced the differentiation of human myeloid leukemia cell line NB-4 cells by ATRA. Then, the polarization of neutrophil-like NB-4 cells to N2-like neutrophils was induced by TGF-*β*. CD11b is an important molecule for neutrophil chemotaxis [38]. In a normal situation, CD11b is mainly stored in intracytoplasmic granules and only expressed at low levels on the cell surface. After neutrophil activation, CD11b expression is upregulated, and it has been found that CD11b can be a characteristic marker of neutrophil activation [39]. To determine the concentration of TGF-*β*, the proportion of CD11b and CD66b (biomarker of neutrophils) was detected via flow cytometer. As result shown, the proportion of CD11b and CD66b was increased with the increase of TGF-*β* concentration at 0.1 and 1 ng/mL. No statistical significance was observed at 1 and 10 ng/mL. The result indicated that, under the concentration of 1 and 10 ng/mL, TGF-*β* activated the neutrophils the best (Figure 2(a)). Thereby, 10 ng/mL TGF-*β* was selected for the subsequence experiment. Interestingly, the proportion was markedly decreased at 20 ng/mL. Also, compared with non-treated neutrophils, the concentration of proinflammatory factors CXCL10 and IL-12 was observed no statistical significance in TGF-*β*-treated neutrophils, while after TGF-*β* treatment, the concentration of anti-inflammatory factors IL-10 and CCL2 was significantly increased, which is consistent with previous notes [25] (Figure 2(b)). Hence, TGF-*β* successfully induced the polarization of neutrophils into N2-like neutrophils. Then, the exosome was extracted from nontreated and N2-like neutrophils. The extracted exosomes were identified via TEM, and small membrane vesicles sized from 40 to 100 nm can be observed (Figure 2(c)). Also, the expression of exosome-related proteins CD63, CD81, TSG101 and Alix was increased in extracted exosomes compared to non-treated and N2-like neutrophils respectively (Figure 2(d)). Using PKH-67 to label exosomes, we observed that exosomes were taken by recipient COLO205 and SW480 (Figure 3(a), *Supplementary 2*). After exosomes were taken up, the aggressive behavior of COLO205 and SW480 was investigated. CCK-8 was used to detect the proliferation of COLO205 and SW480 (Figure 3(b), *Supplementary 2*). Compared with a control group, the proliferation of COLO205 and SW480 was increased significantly after cocultured with exosomes derived from N2-like neutrophils. Also, cell apoptosis was alleviated after the stimulation of exosomes derived from N2-like neutrophils (Figures 3(c) and 3(d), *Supplementary 2*). The results of Wound healing assay and Transwell assay were shown that the migration and invasion of COLO205 and SW480 were promoted by exosomes derived from N2-like neutrophils (Figure 3(e)–3(h), *Supplementary 2*).

The article "miR-4780 Derived from N2-Like Neutrophil Exosome Aggravates Epithelial-Mesenchymal Transition and Angiogenesis in Colorectal Cancer" was retracted in 2023. Reasons: signs of a paper mill; suspected computer-generated content; unreliable results or conclusions; lack of ethics approval or compliance.

### 3.3. miR-4780 Was Enriched in Exosome Derived from Neutrophils and Aggravated EMT and Angiogenesis

Next, the exosomes derived from non-treated (N0-like) and N2-like neutrophils were collected, and microarray was used to find the differential expressed miRNAs in exosomes derived from N2-like neutrophils (Figure 4(a), *Supplementary 1*). According to our previous research [40], two miRNAs (select criteria: *p* < 0.05, fold change >1.5, upregulated) was selected, i.e., hsa-miR-4780 and hsa-miR-513b-3p. Then qPCR was used to verify the expression of miRNAs (Figures 4(b) and 4(c)). The results showed both miRNAs were upregulated in N2-like neutrophils, which is coincident with the results from RNA sequencing. To find EMT-related miRNA, the target genes of hsa-miR-4780 and hsa-miR-513b-3p were predicted and then EMT-related mRNAs were selected according to previous study [38]. We, therefore, chose hsa-miR-4780 for subsequent research. miR-4780 inhibitor and its corresponding negative control vector were transfected into N2-like neutrophils and the exosomes were extracted. CRC cell lines COLO205 and SW480 were cocultured with extracted exosomes. The intake of PKH-67 labeled exosomes was verified with immunofluorescence (Figure 4(d), *Supplementary 2*). The expression of miR-4780 was detected by qPCR. The expression was increased after N2-like neutrophil exosomes stimulation compared with which was cocultured with N0-like neutrophil, while miR-4780 inhibitor reversed the expression (Figure 4(e), Supplementary 2). Also, cocultured with N2-like neutrophil exosome enhanced cell viability and decreased the apoptosis of COLO205 and SW480, while the deprivation of miR-4780 reversed the result (Figures 4(f), 4(g), and 4(j), *Supplementary 2*). Moreover, the ability of migration and invasion was enhanced after cocultured with N2-like neutrophil exosome, while the deprive of miR-4780 reversed the result (Figure 4(h)–4(l), *Supplementary 2*). The expression of EMT associated proteins were also detected via western blot. It is obvious that the expression of E-cadherin was decreased after cocultured with N2-like neutrophil exosome, and the expression of N-cadherin and vimentin was increased, the results were reversed by miR-4780 inhibitor (Figure 5(a)–5(d), Supplementary 2). Therefore, the overexpression of miR-4780 promoted aggressive behavior of COLO205 and SW480 and aggravated metastasis by increasing the incidence of EMT.

To detect the effect of miR-4780 on angiogenesis, we cocultured HUVECs with COLO205 and SW480, and purified neutrophils exosomes were then added. CCK-8 and Wound healing assay were performed to detect the proliferation and migration of HUVECs (Figure 5(e)–5(g), *Supplementary 2*). After the intake of N2-like neutrophil exosome, the proliferation, and migration of HUVECS were increased compared to those with N0-like neutrophil exosomes. While, miR-4780 inhibitor retrieved the result. Also, the tube formation was conducted via BD Matrigel (Figures 5(h) and 5(i), *Supplementary 2*). Similarly, the tube formation was promoted by the intake of N2-like neutrophil exosomes compared with those cocultured with the N0-like neutrophil exosome. The result was retrieved by miR-4780 inhibitor. Also, same trend was observed in the expression of vascular endothelial growth factor (VEGF) and CD34 in HUVECs (Figure 5(j)–5(l), *Supplementary 2*). Hence, N2-like neutrophil exosomal miR-4780 aggravated the angiogenesis by increasing the expression of VEGF and CD34 in HUVECs.

The article "miR-4780 Derived from N2-Like Neutrophil Exosome Aggravates Epithelial-Mesenchymal Transition and Angiogenesis in Colorectal Cancer" was retracted in 2023. Reasons: signs of a paper mill; suspected computer-generated content; unreliable results or conclusions; lack of ethics approval or compliance.

### 3.4. SOX11 Was a Target of miR-4780 and Aggravated EMT and Angiogenesis

The expression of SOX11 was lower expressed in COAD from TCGA (Figure 6(a)). Also, lower expression of SOX11 indicated the favorable overall survival (OS) and disease-free survival (DFS) (Figures 6(b) and 6(c)). Then, the target of miR-4780 was predicted by Target Scan (Ver. 7.2, https://www.targetscan.org/vert_72/), and SOX11 was selected as a target of miR-4780 (Figure 6(d)). To further verify the relationship between miR-4780 and SOX11, dual fluorescence staining is performed (Figure 6(e)). In SOX11 wild-type group, when miR-4780 was overexpressed, relative luciferase activity was decreased. However, there was no significant difference between SOX11 mutate group. We can draw a conclusion that SOX11 was a target of miR-4780.

Next, to evaluate the function of SOX11 in CRC, pcDNA SOX11 was transfected into COLO205 and SW480, which absorbed the extracted exosomes. The expression of miR-4780 and SOX11 was detected via qPCR and western blot (Figure 6(f)–6(h), *Supplementary 2*). The result showed that miR-4780 was highly expressed, while SOX11 was poorly expressed in N2-like neutrophils-derived exosomes. However, the transfection of pcDNA-SOX11 increased the expression. Also, the transfection of pcDNA-SOX11 suppressed the proliferation, migration, and invasion and aggravated the apoptosis of CRC cell lines compared with those only absorbed N2-like neutrophils (*Supplementary 2*). Further, the expression of E-cadherin was increased, and the expression of N-cadherin and vimentin was decreased after pcDNA-SOX11 transfection, which suggested the increase of SOX11 expression suppressed the incidence of EMT (Figure 6(i)–6(l), *Supplementary 2*).

When refers to the effect of SOX11on angiogenesis, the proliferation, migration, and tube formation ability of HUVECS were suppressed after pcDNA-SOX11 transfection compared with those only absorbed N2-like neutrophils (Figure 6(p)–6(s), *Supplementary 2*). The expression of VEGF and CD34 (Figure 6(m)–6(o), *Supplementary 2*) also decreased after pcDNA-SOX11 transfection. Which suggested the increase of SOX11 expression suppressed the incidence of angiogenesis.

The article "miR-4780 Derived from N2-Like Neutrophil Exosome Aggravates Epithelial-Mesenchymal Transition and Angiogenesis in Colorectal Cancer" was retracted in 2023. Reasons: signs of a paper mill; suspected computer-generated content; unreliable results or conclusions; lack of ethics approval or compliance.

### 3.5. miR-4780 Can Aggravate EMT In Vivo

Hepatic metastasis is prevalent in CRC; approximate 35%–55% of patients will develop hepatic metastasis. Thus, we cocultured COLO205 and SW480 with exosomes and injected the cells from teil veins, then investigated the hepatic metastasis in mice. The hepatic metastasis was monitored via *in vivo* live imaging. The hepatic metastasis was aggravated by N2-like neutrophil exosome, which was reversed by miR-4780 inhibitor. (Figure 7(a)) Then, the hepatic function was evaluated by the content of ALT, AST, GGT, and ALP. Obviously, the hepatic function was damaged by N2-like neutrophil exosome, which was reversed by miR-4780 inhibitor (Figure 7(b)). Also, the result of HE staining showed that a larger necrotic area was observed after N2-like neutrophil exosomes stimulation, while miR-4780 inhibitor reversed the result (Figure 7(c)). The expression of miR-4780 and SOX11 in liver tissue was detected. The expression of miR-4780 was increased after N2-like neutrophil exosomes stimulation compared with which was cocultured with N0-like neutrophil, while miR-4780 inhibitor reversed the expression (Figures 7(d) and 7(e)). Also, the expression of SOX11 was decreased after cocultured with N2-like neutrophil exosome, while the results was reversed by miR-4780 inhibitor. The expression of EMT-relative proteins in liver tissue was detected by western blot and immunofluorescence (Figures 7(f), 7(g), 7(i), and 7(j)). The results showed that the expression of epithelial surface makers (i.e., E-cadherin and occludin) was decreased by N2-like neutrophil exosome, while the expression of mesenchymal makers (i.e., N-cadherin, vimentin, and Zo1) was increased. Also, the expression of CD34 and VEGF was increased by N2-like neutrophil exosome (Figures 7(h), 7(k), and 7(l)). However, the deprive of miR-4780 reversed the expression, which indicated that miR-4780 derived from N2-like neutrophil exosome aggravated EMT and angiogenesis (Figure 8).

## 4. Discussion

In this study, we first verified the enrichment of neutrophils in tumor tissues harvested from CRC, and the expression of CD11b is correlated with tumor site and the presence of invasion of serosa. Also, we proved that the internalization of N2 exosomes aggravated the viability, migration, and invasion of CRC cell lines and suppressed the cell apoptosis. To further investigate the molecular mechanism, we conducted the miRNA expression profile in the N2-like neutrophils and thereby choose hsa-miR-4780 for a subsequent experiment. We found that the overexpression of miR-4780 from N2-like neutrophil-derived exosome aggravated the EMT and angiogenesis. Moreover, miR-4780 can regulate its target gene SOX11 to affect the EMT and angiogenesis of CRC cell lines. CRC with liver metastasis model also verified that abnormal expression of miR-4780 from N2-like neutrophil-derived exosome aggravated the metastasis and development of tumor via EMT and angiogenesis.

The article "miR-4780 Derived from N2-Like Neutrophil Exosome Aggravates Epithelial-Mesenchymal Transition and Angiogenesis in Colorectal Cancer" was retracted in 2023. Reasons: signs of a paper mill; suspected computer-generated content; unreliable results or conclusions; lack of ethics approval or compliance.

The presence of neutrophils in tumors has traditionally been regarded as indicative of a failed immune response against cancer [41]. However, recent reports have revealed multiple roles for neutrophils besides immune response signaling. In this manuscript, the analyzed result from TCIA showed that neutrophils are relatively enriched in CRC and is one of the most infiltrated immune cells (approximately 32%). Also, neutrophils were enriched in the tumor tissues we harvested from primary CRC patients. The relationship between TAN and human cancer has not been systemically investigated, although the increase of neutrophils counts in peripheral blood, also known as neutrophils-to-lymphocyte ratio (NLR), has been regarded as a poor prognostic factor in CRC [42]. Ashizawa et al. [43] showed that decreasing post-NLR was related to a better OS rate and DFS even in high pre-NLR patients with CRC. Li et al. [44] retrospectively analyzed a cohort of 354 CRC patients and revealed that the NLR was an independent prognostic factor for OS in early-stage colon cancer. Ye et al. [33] also proved that the number of CD66b^+^ TANs, Tregs, and TAMs were more reliable than traditional indicators for evaluating prognosis in CRC patients. In this manuscript, we found that the expression of CD11b is correlated with tumor site and the presence of invasion of serosa. Many lineages of stromal cells contained in TEM have been reported to promote the growth of CRCs, including TAN. Intriguingly, the role of neutrophils in tumor growth and metastasis was controversial. This can be explained by the phenotypically plastic of neutrophils with similarities to corresponding macrophage populations [27]. Accumulated results suggested that tumors can induce a pro-tumor phenotype in neutrophils that, in turn, help tumor progression. Raccosta et al. [45] have shown that oxysterol derived from tumor cells recruit protumor neutrophils, thus favoring tumor growth by promoting neoangiogenesis and immunosuppression. Fridlender et al. [25] showed that TGF-*β* within the TME induces the phenotypically plastic of neutrophils and increased the activation and population of TAN with a protumor phenotype. Neutrophil elastase and prostaglandin E2 secreted by neutrophils are proved to promote tumor cell proliferation [46, 47]. In line with these results, we found that exosomes derived from TGF-*β* induced N2-like neutrophils can also promote the growth of CRC.

The article "miR-4780 Derived from N2-Like Neutrophil Exosome Aggravates Epithelial-Mesenchymal Transition and Angiogenesis in Colorectal Cancer" was retracted in 2023. Reasons: signs of a paper mill; suspected computer-generated content; unreliable results or conclusions; lack of ethics approval or compliance.

Metastasis is the primary contributor to death in patients with solid cancers. Largely due to our poor understanding on the cellular and molecular process associated with metastasis, once the tumor has spread from the primary site, neither conventional chemotherapy nor current targeted therapy offers significant benefits [48]. Despite that CRC is the result of multiple factors, metastasis is an important factor that affects the survival and prognosis of CRC. At least one-third of CRC patients develop liver metastases [49]. Reports show that the 5-year survival rate of patients with early CRC can reach more than 90%, while the rate drops to 69.2% for patients with local metastasis and less than 10% for patients with distant metastasis [50]. EMT is a cellular process in which cell lost their epithelial characteristics and acquire mesenchymal features [51]. EMT has been reported to be involved in various tumor functions, including tumor initiation, malignant progression, tumor stemness, tumor cell migration, intravasation to the blood, metastasis, and resistance to therapy. Li et al. [52] proved that TANs produce IL-17a and promote EMT of GC cells via JAK2/STAT3 signaling. Likewise, Zhang et al. [24] proved that interaction with neutrophils aggravated the migration and invasion through the activation of the ERK pathway and the induction of EMT in gastric cancer. Angiogenesis is a critical step not only in tumor development but in distant metastases. Accumulated results suggested that except tumor cells, stromal cells in the TME also participated in the process of angiogenesis. Neutrophils recruited to malignant site produces matrix metalloproteinase-9 and VEGF and therefore participates in the incidence of angiogenesis [53]. Shojaei et al. [54] showed that BV-8 overexpression modulates the mobilization of CD11b^+^Gr1^+^ neutrophils and therefore promotes angiogenesis. Consistent with these results, we found hsa-miR-4780 in exosome derived by N2-like neutrophils promote EMT and angiogenesis in CRC.

SOX11 is a member of sex-determining region Y-related a high mobility group-box (SOX) family, which are characterized as transcription factors with a high mobility group (HMG) DNA-binding domain [55]. Based on the protein sequence alignment, the SOX gene family was divided into 10 groups from A to J. SOX11, together with SOX4 and SOX12 are members of subgroup C, which bind to the 5′-(A/T) (A/T) CAA(A/T) G-3′ consensus site, and thus induce several DNA conformational changes that allow other transcription factors/regulatory proteins to bind together [56]. Similar to SOX4, SOX11 has been reported to be essential for organogenesis, neurodevelopment, and neuronal growth. Recently, SOX11 was reported as a key oncogenic factor in mantle cell lymphoma. Moreover, SOX11 and its hypermethylation were reported to be involved in the progression of head and neck cancer [57], cervical cancer [58], prostate cancer [59], etc. Wang et al. [60] proved that miR-31 modulates EMT in papillary thyroid carcinoma by targeting SOX11. Likewise, SOX11 was reported to promote angiogenesis in mantle cell lymphoma [61, 62]. However, other reports have shown that SOX11 plays an oncogenic role in small-cell lung cancer [63] and acute myeloid leukemia [64]. This suggests that the differential role of SOX11 in tumors may be related to tissue specificity and TME. In this manuscript, we found that hsa-miR-4780 in exosome derived by N2-like neutrophils promotes EMT and angiogenesis by targeting SOX11 in CRC.

The article "miR-4780 Derived from N2-Like Neutrophil Exosome Aggravates Epithelial-Mesenchymal Transition and Angiogenesis in Colorectal Cancer" was retracted in 2023. Reasons: signs of a paper mill; suspected computer-generated content; unreliable results or conclusions; lack of ethics approval or compliance.

However, there are also some limitations existed in this manuscript. The limited number of patient samples due to difficulties in tissue collection, especially in tumor tissue from patients with distant metastases, may account for the lack of correlation found between CD66b and clinicopathological parameters. Circulating tumor cells (CTCs), which are shed from primary or secondary tumors and actively invade the bloodstream, are regarded as one of the predominant factors for distant metastases [65, 66]. Wei et al. [67] indicated that tumor-associated macrophages-induced EMT programs can enhance the migration and invasion of CTCs, and in turn promote macrophage recruitment. Whether similar crosstalk can be validated between CTCs and N2-like TAN deserves further investigation.

In conclusion, for the first time, our current finding discloses an important mechanism that mR-4780 from N2-like neutrophil-derived exosome aggravated the metastasis and development of tumor via EMT and angiogenesis.

## Figures and Tables

**Figure 1:** Neutrophils are enriched in colorectal cancer tissue. (a) Gene set enrichment analysis in various cancer via cancer immunome database (TCIA, https://tcia.at/home). (b) The fraction of immune cell profile in tumor microenvironment (TEM) of CRC. (c and d) Immunohistochemistry staining and percentage of positive cells of CD66b in CRC tumor tissues and their corresponding para-cancerous tissues (×40). (e and f) Immunohistochemistry staining and percentage of positive cells of CD11b in 30 CRC tumor tissues and their corresponding para-cancerous tissues (×40). Error bars represent SD.  ^*∗∗∗∗*^*p* < 0.0001. *n* = 30.

The article "miR-4780 Derived from N2-Like Neutrophil Exosome Aggravates Epithelial-Mesenchymal Transition and Angiogenesis in Colorectal Cancer" was retracted in 2023. Reasons: signs of a paper mill; suspected computer-generated content; unreliable results or conclusions; lack of ethics approval or compliance.

**Figure 2:** Neutrophils polarization and exosome verification. (a) The proportion of CD11b and CD66b was detected via flow cytometer. (b) The concentration of proinflammatory factors CXCL10 and IL-12 and anti-inflammatory factors IL-10 and CCL2 was detected via ELISA. (c) Representative TEM image of morphology of BMSCs released exosomes. Scale bar = 1 *μ*m. (d) The expression of exosomes section-associated protein was detected. Error bars represent SD.  ^*∗∗∗*^*p* < 0.001;  ^*∗∗∗∗*^*p* < 0.0001.

**Figure 3:** Exosomes derived from N2-like neutrophils promote the tumor progression of COLO205. (a) Exosomes were labeled by PKH-67 (green), and the internalization of exosomes by COLO205 was observed (×40). (b) CCK8 assay for cellular viability. (c and d) Cell apoptosis was detected by flow cytometer. (e and f) Wound healing assay for cell migration (×10). (g and h) Transwell assay for cell invasion (×10). Error bars represent SD.  ^*∗*^*p* < 0.05;  ^*∗∗*^*p* < 0.01;  ^*∗∗∗*^*p* < 0.001;  ^*∗∗∗∗*^*p* < 0.0001.

**Figure 4:** miR-4780 was enriched in exosome derived from neutrophils and promotes the tumor progression of COLO205. (a) The hierarchic clustering of differentially expressed miRNAs was plotted to show a distinguishable miRNA expression profiling between N0-exo and N2-exo. Red represents relatively high expression; green represents relatively low expression. (b and c) miR-4780 and miR-513b-3p were both highly expressed in N2-exo. (d) Exosomes were labeled by PKH-67 (green), and the internalization of exosomes by COLO205 was observed. (e) Expression of miR-4780 in exosomes was measured via qPCR. (f and g) Cell apoptosis was detected by flow cytometer. (h and i) Wound healing assay for cell migration (×10). (j) CCK8 assay for cellular viability. (k and l) Transwell assay for cell invasion (×10). Error bars represent SD.  ^*∗*^*p* < 0.05;  ^*∗∗*^*p* < 0.01;  ^*∗∗∗∗*^*p* < 0.0001.

**Figure 5:** miR-4780 promotes the EMT and angiogenesis of COLO205. (a–d) The expression of EMT-associated proteins, E-cadherin, N-cadherin, and vimentin in COLO205 were measured via western blot. (e) CCK8 assay for cellular viability of HUVECs. (f and g) Wound healing assay for cell migration of HUVECs (×10). (h and i) Tube formation assay was conducted, and the tube number was calculated (×40). (j–l) The expression of angiogenesis-associated proteins, CD34 and VEGF in HUVECs were measured via western blot. Error bars represent SD.  ^*∗*^*p* < 0.05;  ^*∗∗*^*p* < 0.01;  ^*∗∗∗*^*p* < 0.001;  ^*∗∗∗∗*^*p* < 0.0001.

The article "miR-4780 Derived from N2-Like Neutrophil Exosome Aggravates Epithelial-Mesenchymal Transition and Angiogenesis in Colorectal Cancer" was retracted in 2023. Reasons: signs of a paper mill; suspected computer-generated content; unreliable results or conclusions; lack of ethics approval or compliance.

**Figure 6:** SOX11 was a target of miR-4780 and aggravated EMT and angiogenesis of COLO205. (a) The expression of SOX11 in COAD from TCGA. (b and c) Overall survival and disease-free survival of SOX11 in COAD from TCGA. (d) Structure of human SOX11 gene and location of hsa-miR-4780. (e) Relative luciferase activity of different groups. (f) Expression of miR-4780. (g and h) Protein expression of SOX11. (i–l) The expression of EMT-associated proteins, E-cadherin, N-cadherin, and vimentin in COLO205 were measured via western blot. (m–o) The expression of angiogenesis-associated proteins, CD34, and VEGF in HUVECs were measured via western blot. (p) CCK8 assay for cellular viability of HUVECs. (q–s) Wound healing assay for cell migration of HUVECs. (n, p; ×10) and tube formation assay (o, q; ×40)  ^*∗*^*p* < 0.05;  ^*∗∗*^*p* < 0.01;  ^*∗∗∗∗*^*p* < 0.0001.

**Figure 7:** miR-4780 can aggravated EMT *in vivo*. (a) Represent images of *in vivo* bioluminescence imaging of tumor growth. (b) The content of ALT, AST, GGT, and ALP in liver tissue. (c) He staining in liver tissue. (d) Protein expression of SOX11 in liver tissue. (e) Expression of miR-4780 in liver tissue. (f) The expression of EMT-associated proteins, E-cadherin, N-cadherin, vimentin, and occludin in liver tissue. (g) Immunofluorescence staining of ZO-1 and vimentin. (×40) (h) Immunohistochemical staining for CD34 and VEGF. Error bars represent SD (×40). (i, j) Mean fluorescence of ZO-1 and vimentin. (k, l) Positive area of CD34 and VEGF.  ^*∗*^*p* < 0.05;  ^*∗∗*^*p* < 0.01;  ^*∗∗∗*^*p* < 0.001;  ^*∗∗∗∗*^*p* < 0.0001. *n* = 10.

**Figure 8:** miR-4780 derived from N2-like neutrophil exosome aggravated EMT and angiogenesis. Exosome derived from neutrophils was extracted, and differentially expressed miRNA in neutrophils-derived exosomes has been sequenced by microarray profile. In this manuscript, we found that hsa-miR-4780 in exosome derived by N2-like neutrophils promotes EMT and angiogenesis by targeting SOX11 in the colorectal cancer.

**Table 1:** Primary antibodies used in western blot.

Primary	Company	Catalog number	Dilution
Alix	Abcam	ab88388	1 : 1,000
CD63	Abcam	ab134045	1 : 1,000
CD81	Abcam	ab109201	1 : 1,000
TSG101	Abcam	ab125011	1 : 1,000
SOX11	Abcam	ab170916	1 : 1,000
E-cadherin	Abcam	ab40772	1 : 5,000
N-cadherin	Abcam	ab76011	1 : 1,000
Vimentin	Abcam	ab92547	1 : 1,000
CD34	Abcam	ab81289	1 : 10,000
VEGF	Abcam	ab32152	1 : 1,000
Occludin	Abcam	ab216327	1 : 1,000
GADPH	Abcam	P30008M	1 : 1,000

**Table 2:** Correlation between the density of neutrophils at tumor tissue and clinicopathologic parameters (*n* = 30).

Parameter	*n* (%)	CD66b expression			CD11b expression		
		Low	High	*P*	Low	High	*P*
		*n* (%)	*n* (%)		*n* (%)	*n* (%)	
Gender				0.156			0.411
Male	16 (53.33)	4 (33.33)	12 (66.67)		8 (66.67)	8 (44.44)	
Female	14 (46.67)	8 (66.67)	6 (33.33)		4 (33.33)	10 (55.56)	
Age, years				0.693			0.693
<60	10 (33.33)	5 (41.67)	5 (27.78)		3 (25.00)	7 (38.89)	
≧60	20 (66.67)	7 (58.33)	13 (72.22)		9 (75.00)	11 (61.11)	
Tumor site				0.901			0.059^*∗*^
Ileocecum	4 (13.33)	2 (16.67)	2 (11.11)		2 (16.67)	2 (11.11)	
Left colon	16 (53.33)	6 (50.00)	10 (55.56)		9 (75.00)	7 (38.89)	
Right colon	10 (33.33)	4 (33.33)	6 (33.33)		1 (8.33)	9 (50.00)	
Tumor diameter				0.142			0.104
<5 cm	11 (36.67)	2 (16.67)	9 (50.00)		7 (58.33)	4 (22.22)	
≧5 cm	19 (63.33)	10 (83.33)	9 (50.00)		5 (41.67)	14 (77.78)	
Tumor grade				1.00			0.599
Poor	13 (43.33)	5 (41.67)	8 (44.44)		4 (33.33)	9 (50.00)	
Moderated/well	17 (56.67%)	7 (58.33)	10 (55.56)		8 (66.67)	9 (50.00)	
TNM stage^a^				0.935			1.00
I and II	21 (70.00)	9 (75.00)	12 (66.67)		8 (66.67)	13 (72.22)	
III and IV	9 (30.00%)	3 (25.00)	6 (33.33)		4 (33.33)	5 (27.78)	
LNM				1.00			1.00
Presence	7 (23.33)	3 (25.00)	4 (22.22)		3 (25.00)	4 (22.22)	
Absence	23 (76.67)	9 (75.00)	14 (77.78)		9 (75.00)	14 (77.78)	
Invasion of serosa				1.00			0.040^*∗*^
Presence	18 (60.00)	7 (58.33)	11 (61.11)		4 (33.33)	14 (77.78)	
Absence	12 (40.00)	5 (41.67)	7 (38.89)		8 (66.67)	4 (22.22)	
Total	30 (100)	12 (100)	18 (100)		12 (100)	18 (100)	

^a^The 8th edition of the AUCC Cancer Staging Manual.  ^*∗*^*P* < 0.05. LNM, lymph node metastasis; TNM, tumor-node-metastasis; CD66, cluster of differentiation of 66; CD11b, cluster of differentiation of 11b. Bold values signify statistical significance.

The article "miR-4780 Derived from N2-Like Neutrophil Exosome Aggravates Epithelial-Mesenchymal Transition and Angiogenesis in Colorectal Cancer" was retracted in 2023. Reasons: signs of a paper mill; suspected computer-generated content; unreliable results or conclusions; lack of ethics approval or compliance.

## Data Availability

All data, models, or code generated or used during the study are available from the corresponding author by request.

## Supplementary Materials

Supplementary 1 Clinical characteristics of patients (*n* = 30). Differential expressed miRNAs.

Supplementary 2 Exosomes derived from N2-like neutrophils promote the tumor progression of SW480. miR-4780 promotes the tumor progression of SW480. miR-4780 promotes the EMT and angiogenesis of SW480. SOX11 promotes the tumor progression of COLO205. SOX11 was a target of miR-4780 and aggravated EMT and angiogenesis of SW480.
